This article has been retracted.

# CircEIF4G2 Promotes Tumorigenesis and Progression of Osteosarcoma by Sponging miR-218

**DOI:** 10.1155/2020/8386936

**Published:** 2020-05-23

**Authors:** Erhu Lin, Shuai Liu, Wei Xiang, Hongbo Zhang, Chaofan Xie

**Affiliations:** ^1^Spinal Surgery Department, Shenzhen People's Hospital, Shenzhen, Guangdong 518000, China; ^2^Orthopedics Department, The Eight Affiliated Hospital of Sun Yat-sen University, Shenzhen, Guangdong 518000, China

## Abstract

Circular RNAs (circRNAs) play a key role in regulating the tumorigenesis and development of human cancers, including osteosarcoma (OS). Of note, the molecular mechanism underlying the progression of OS has remained largely unclear. The present study identified that a novel circRNA circEIF4G2 was upregulated in OS tissues and cells. Moreover, we constructed a circEIF4G2-mediated ceRNA network and revealed that circEIF4G2 was involved in regulating multiple cancer pathways, such as the EGFR signaling pathway, the PI3K-Akt signaling pathway, and the ErbB signaling pathway. Loss-of-function assays showed that circEIF4G2 knockdown significantly suppressed OS cell proliferation, migration, and invasion. Mechanically, we found that circEIF4G2 could directly bind to miR-218, and miR-218 mediated the effect of circEIF4G2 knockdown on OS progression. In conclusion, the present study showed that circEIF4G2 could be a potential biomarker for OS.

## 1. Introduction

Osteosarcoma (OS) is one of the most common bone malignancies originating from active regions in the bone occurring in adolescents [1]. Over the past decades, multiple genomic factors were revealed to be related to OS, including miRNAs [2], lncRNAs [3], and transcription factors [4]. For instance, miR-627-3p was reported to inhibit OS cell proliferation by reducing PTN [5], and miR-548d-3p was reported to inhibit OS by downregulating KRAS [6]. lncRNA TUG1 could promote OS cell metastasis by mediating HIF-1*α* [7] and AKT signaling [8]. However, treatment of advanced-stage OS was still a challenge. Therefore, it is still an urgent need to explore novel therapeutic biomarkers for OS.

Increasing studies demonstrated that circular RNAs (circRNAs) were widespread in human cells [9, 10]. circRNAs were a special class of noncoding RNAs which has a characteristic loop structure without 5′ or 3′ ends [11]. Emerging studies have shown that circRNAs play a crucial role in regulating cell growth, cell cycle, cell apoptosis, cell migration, and cell metabolism in a series of cancer types, including OS [12]. For example, Pan et al. found that circMMP9 promotes OS progression via targeting the miR-1265/CHI3L1 axis [13]. Zheng et al. found that circRNA LRP6 induced OS development via negatively regulating KLF2 expression [14]. Mechanically, circRNAs were confirmed to regulate gene expression through binding to miRNAs. circRNA CDR1as was reported to be a miR-7 sponge in nasopharyngeal carcinoma [15], hepatocellular carcinoma [16], ovarian cancer [17], non-small-cell lung cancer [18], and OS [19].

EIF4G2 was reported to be an oncogene in OS [20]. Knockdown of EIF4G2 suppressed OS proliferation, migration, and invasion [20]. However, the molecular functions and mechanisms of circEIF4G2 in OS remained unclear. The point of the present study is exploring the roles of circEIF4G2 in OS.

## 2. Materials and Methods

### 2.1. Osteosarcoma Specimens

There were 62 OS and 13 normal tissues in total collected from our hospital, and this study was reviewed and approved by the Ethics Committee. The acquisition of the human samples involved in this study was in compliance with the ethical and legal standards, and the patients involved gave informed consent.

### 2.2. Cell Culture and Cell Transfection

HOS and MG63 were cultured in complete DMEM medium, which is based on basal DMEM medium (HyClone, Logan, UT, USA) mixed with 10% fetal bovine serum (FBS) and 100 U/mL of penicillin/streptomycin double antibiotics. The sequences were as follows: si-circEIF4G2, 5′-AUGCUCCCAGCUUUUGGAAAA-3′; si-NC, 5′-UUCUCCGAACGUGUCACGU-3′; miR-218 mimic, 5′-UUGUGCUUGAUCUAACCAUGU-3′; miR-NC, 5′-UUCUCCGAACGUGUCACGU-3′; and miR-218 inhibitor, 5′-ACAUGGUUAGAUCAAGCACAA-3′.

### 2.3. CCK-8 Assay

Cell proliferation was detected and calculated using the CCK-8 assay according to previous studies [21].

### 2.4. Cell Invasion Assay

The Transwell chambers were placed into a 24-well plate. The space in the Transwell chambers was called the upper compartment. The space between the Transwell chambers and the culture plate was called the lower compartment. They were separated by filters. 30 *μ*L Matrigel was coated on the upper surface of the filters. And 50,000 cells in 200 *μ*L of serum-free DMEM were seeded in the upper compartment, while 600 *μ*L of DMEM containing 10% FBS was added to the lower compartment. The cell invasion ability was reflected by the number of cells which passed through the filter, was fixed with formaldehyde, and was stained with crystal violet at the bottom of the filter.

### 2.5. qRT-PCR

Total RNA from the HOS, MG63, and patient's samples was extracted using the TRIzol Reagent, and then RNA concentration was quantified by 260 nm/280 nm. A moderate amount of RNA was used for reverse transcription according to the instructions of the reverse transcription kit (TaKaRa, Shiga, Japan). The cDNA was mixed with SYBR Premix Ex Taq II (TaKaRa, Shiga, Japan), primers, and H_2_O, and the cycle threshold (Ct) of the mixture was detected. The expression of 18S rRNA (18S) was used to calibrate the expression of the target genes through the 2^-ΔΔCt^ method. Calibration according to U6 and miR-218 were quantified by the Hairpin-it miRNA qPCR Quantitation Kit (Shanghai GenePharma Co., Ltd.). The primers used in this study included circEIF4G2 5′-TTTTTCAACAAAGCAAGGTCAA-3′ and 5′-TCTAGGTCCCACTGTCCTCA-3′, miR-218 5′-CGCGCGCGTTGTGCTTGATCTAA-3′ and 5′-AGTGCAGGGTCCGAGGTATT-3′, GAPDH 5′-GTGTTTCCTCGTCCCGTAGA-3′ and 5′-GAATTTGCCGTGAGTGGAGT-3′, and U6 5′-GCTTCGGCAGCACATATACTAAAAT-3′ and 5′-TACTGTGCGTTTAAGCACTTCGC-3′.

### 2.6. Dual-Luciferase Reporter Assay

Dual-luciferase reporter assay was assessed by the Dual-Luciferase Reporter Assay System (Promega Corporation, Madison, WI, USA). The cells were cotransfected with two plasmids and then cleaved after 48 h. Substrates were added to the cell lysates. The relative luciferase signal was presented as firefly luciferase activity normalized to renilla luciferase activity. The ability of miRNA binding to circEIF4G2 was reflected by the relative luciferase signal of firefly luciferase normalized to renilla luciferase. To construct the recombinant luciferase vectors, wild-type (WT) and mutant (MUT) circEIF4G2 sequences were synthesized by Shanghai GenePharma Co., Ltd. (Shanghai, China) and separately cloned into pmirGLO luciferase vectors (Promega Corporation, Madison, WI, USA) between the NheI and XbaI sites. In addition, WT and MUT 3′-UTRs of HOXA1 were synthesized by Shanghai GenePharma Co., Ltd. and separately cloned into pmirGLO luciferase vectors between the SacI and XbaI sites. HeLa or C33A cells were cotransfected with 50 nM miR-218 mimic or miR-NC, and the recombinant luciferase vectors using Lipofectamine® 3000 (Invitrogen; Thermo Fisher Scientific, Inc.). After 48 h of incubation, luciferase activity was detected using the Dual-Luciferase Reporter Assay System (Promega Corporation) according to the manufacturer's protocol. Renilla luciferase activity was detected and used as the internal control.

### 2.7. Construction of the ceRNA Network

The Circular RNA Interactome (https://circinteractome.nia.nih.gov/) and Cancer-Specific circRNA Databases (http://gb.whu.edu.cn/CSCD/) were used to predict the regulatory relationships between circRNAs and miRNAs. The circRNA-miRNA-mRNA network was established using a combination based on circRNA-miRNA pairs and miRNA-mRNA pairs and was visualized using Cytoscape software (version 3.7.0; http://cytoscape.org/).

### 2.8. Functional Enrichment Analysis

Gene Ontology (GO) and Kyoto Encyclopedia of Genes and Genomes (KEGG) analyses were conducted using the Cluster Profiler package (version 3.12.0) of R software (version 3.6.1; http://www.r-project.org), in order to assess the primary function of the DEmRNAs in the ceRNA network in tumorigenesis.

### 2.9. Statistical Analysis

The data in the study were subjected to at least three separate experiments, which were visualized by a column diagram with mean and standard deviation (SD). One-way ANOVA or Student's t-test was used to detect whether the difference between groups was significant by SPSS 20.0 software (IBM, NY, USA). The P value < 0.05 was considered statistically significant.

## 3. Results

### 3.1. CircEIF4G2 Was Upregulated in OS

In order to validate the upregulation of circEIF4G2 in OS, we detected its expression levels in OS samples. qRT-PCR analysis results indicated that the expression of circEIF4G2 was significantly higher in osteosarcoma tissues than in normal tissues (Figure 1(a), p < 0.05). Moreover, overexpression of circEIF4G2 was also present in osteosarcoma HOS and MG63 cell lines compared to hFOB1.19 cells (Figure 1(b)).

### 3.2. CircEIF4G2 Affects Osteosarcoma Cell Viability, Invasion, Migration, and Apoptosis

CircEIF4G2 was significantly downregulated in HOS (Figure 1(c)) and MG63 (Figure 1(d)) cells after knockdown of circEIF4G2. The CCK-8 assay showed that circEIF4G2 knockdown significantly suppressed HOS (Figure 2(a)) and MG63 (Figure 2(b)) cell growth, and the Transwell assay revealed that circEIF4G2 knockdown remarkably reduced the cell migration (Figure 2(c)) and invasion (Figure 2(e)) of HOS cells compared with the control group. Very interestingly, we observed a similar result in MG63 cells (Figures 2(d) and 2(f)).

### 3.3. Construction of CircEIF4G2-Mediated ceRNA Networks in OS

Of note, we further conducted bioinformatics analysis to identify circEIF4G2-mediated ceRNA networks in OS. We used the RegRNA 2.0 database (http://regrna2.mbc.nctu.edu.tw/index.html) [22] to predict circEIF4G2-miRNA interaction and used the starBase v2.0 database to predict miRNA-mRNA interaction. As presented in Figure 3, a total of 5 miRNAs (hsa-miR-218-5p, hsa-miR-188-5p, hsa-miR-4465, hsa-miR-517-5p, and hsa-miR-525-5p) and 2187 mRNAs were included in this ceRNA network.

### 3.4. Bioinformatics Analysis of CircEIF4G2 in OS

Next, we conducted bioinformatics analysis of circEIF4G2 using its potential ceRNA targets using the DAVID system. GO analysis showed that circEIF4G2 was involved in the regulation of the EGFR signaling pathway; in the regulation of transcription, covalent chromatin modification, and protein phosphorylation; in the positive regulation of cell proliferation, signal transduction, G2/M transition of mitotic cell cycle, actin cytoskeleton reorganization, fibroblast growth factor receptor signaling pathway, endochondral ossification, intracellular signal transduction, transforming growth factor beta receptor signaling pathway, nervous system development, peptidyl-threonine phosphorylation, and peptidyl-serine phosphorylation; in the positive regulation of the ER-associated ubiquitin-dependent protein catabolic process; and in the negative regulation of epidermal growth factor receptor signaling pathway, outer ear morphogenesis, axonogenesis, and protein polyubiquitination (Figure 4(a)).

The KEGG pathway analysis showed that circEIF4G2 was related to endocytosis, estrogen signaling pathway, Rap1 signaling pathway, chronic myeloid leukemia, neurotrophin signaling pathway, sphingolipid signaling pathway, chemokine signaling pathway, melanogenesis, PI3K-Akt signaling pathway, viral carcinogenesis, oxytocin signaling pathway, and ErbB signaling pathway (Figure 4(b)). There results suggested that circEIF4G2 may serve as a key regulator in OS progression.

### 3.5. CircEIF4G2 Sponges miR-218

Among the 5 potential circEIF4G2-targeting miRNAs, miR-218 had been reported to be a direct target of circEIF4G2 by Mao et al. miR-218 played as a tumor suppressor in multiple human cancers. Dual-luciferase reporter assay showed that miR-218 was also a direct target of circEIF4G2 in both HOS and MG63 cells. Compared with the mutant plasmids, miR-218 decreased the relative luciferase activity of the wild-type circEIF4G2 luciferase plasmid significantly (Figures 5(a) and 5(b), p < 0.05).

### 3.6. Effects of miR-218 on Osteosarcoma Cells

Considering that the detailed molecular functions of miR-218 in OS remained unclear, we conducted a gain-of-function assay in OS cells. As shown in Figure 5, after miR-218 was transfected into MG63 and HOS cells, cell proliferation (Figures 5(c) and 5(d)), migration (Figures 5(e) and 5(g)), and invasion (Figures 5(f) and 5(h)) were significantly suppressed compared to the control group.

### 3.7. Silencing of miR-218 Reverses the Effects of CircEIF4G2 Knockdown in OS

The effects of circEIF4G2 knockdown cells including decreased cell proliferation (Figures 6(a) and 6(b)), migration (Figure 6(c)), invasion (Figure 6(d)) were reversed by silencing of miR-218.

## 4. Discussion

The eukaryotic translation initiation factor 4, *γ* (EIF4G) is expressed in mammalian cells in two forms, namely, EIF4G1 and EIF4G2 [23, 24]. Emerging studies demonstrated that disrupted translational machinery strongly contributes to cancer development and progression [25]. EIF4G2 was reported to be an oncogene in multiple human cancers, such as non-small-cell lung cancer (NSCLC) [26] and OS [20]. As lung cancer remains the leading cause of cancer-related deaths [27, 28], understanding the underlying molecular mechanism of NSCLC is desired; EIF4G2 is known to participate in the regulation of cisplatin (CDDP) resistance [26]. In OS, knockdown of EIF4G2 significantly decreased translation and cell proliferation and induced cellular senescence [20]. The circRNA isoform of EIF4G2 was found to be upregulated in cervical cancer (CC) [29]. The molecular function studies demonstrated that circEIF4G2 acted as an oncogene in CC by promoting cell proliferation. However, the roles of circEIF4G2 in OS remain unclear.

The present study first detected the expression of circEIF4G2 in OS samples. Our results showed that circEIF4G2 was upregulated in both OS tissues and cells compared to normal samples and cell lines, suggesting that circEIF4G2 may play a crucial role in the development of OS. Furthermore, cell function assays were performed in vitro. In HOS and MG63, cell proliferation, migration, and invasion were suppressed by knocking down circEIF4G2. These results showed that circEIF4G2 plays an oncogenetic role in promoting the tumorigenesis of OS, which is consistent with previous studies.

Bioinformatics analysis was a powerful tool to understand the potential roles of novel circRNAs in OS [30]. The present study showed that circEIF4G2 was widely involved in regulating multiple pathways, such as the EGFR signaling pathway, the PI3K-Akt signaling pathway, and the ErbB signaling pathway. The ErbB receptor family including EGFR, HER2, HER3, and HER4, played a key role in activating PI3K/Akt and MAPK signaling [31]. Previous studies had demonstrated that ErbB signaling regulated cancer proliferation and metastasis [31]. In OS, ErbB signaling was also revealed to be overexpressed and activated in cancer cells [32, 33]. Targeting ErbB signaling had been a potential therapeutic strategy in OS.

miRNAs are a type of small RNAs with 22 nucleotides, which play a key role in regulating cancer growth, metastasis, and glycolysis by modulating gene expression at the posttranscriptional level [34]. Recently, multiple studies showed that circRNAs played their roles in cancer cells by acting as competing endogenous RNAs (ceRNAs) to sponge miRNAs. For example, circ-AKT3 was found to suppress clear cell renal cell carcinoma metastasis via miR-296-3p/E-cadherin [35]. circRNA_100269 was reported to suppress gastric cancer growth by targeting miR-630 [36]. Circular RNA_LARP4 was reported to suppress gastric cancer cell proliferation and invasion by sponging miR-424-5p [37]. CircEIF4G2 was found to promote CC progression through sponging miR-218 to upregulate HOXA1 [29]. The present study also evaluates the mechanisms of circEIF4G2 underlying OS progression. Using bioinformatic methods, we identified that circEIF4G2 could target miR-218. miR-218 was reported to be a tumor suppressor in OS cells by suppressing E2F2 [38], BIRC5 [39], TIAM1 [40], MMP2 [40], and MMP9 [40]. Dual-luciferase reporter assay showed that circEIF4G2 directly binds to miR-218. Overexpression of miR-218 suppressed circEIF4G2 levels. Moreover, knockdown of miR-218 reversed the decreased cell proliferation, migration, and invasion in cell knockdown of circEIF4G2. miR-218 was reported to be a tumor suppressor in multiple human cancers, including cervical cancer, gliomas, prostate cancer, and colon cancer. For example, miR-218 promotes apoptosis of SW1417 human colon cancer cells by targeting c-FLIP, inhibiting the proliferation of human glioma cells through the downregulation of Yin Yang 1 and inhibiting tumor angiogenesis via targeting the mTOR component RICTOR in prostate cancer.

In this study, there also existed some limitations. Firstly, more samples were needed considering the small sample size in the present study. Secondly, we think that further experimental validation in vivo would be required for future verification. Thirdly, gain-of-function assays should be conducted to validate the roles of circEIF4G2.

In conclusion, this study reported that circEIF4G2 promotes OS tumorigenesis and progression by sponging miR-218. We thought our investigation provided a novel biomarker for OS prognosis and treatment.

## Figures and Tables

**Figure 1:** CircEIF4G2 was upregulated in OS. (a) CircEIF4G2 expression in OS tissues was higher than that in normal tissue. (b) CircEIF4G2 expression was upregulated in OS cells. (c and d) CircEIF4G2 expression levels were reduced in MG63 and HOS after transfecting with siRNAs against circEIF4G2. ^∗^p < 0.05.

**Figure 2:** Effects of circEIF4G2 on OS cell viability, migration, and invasion ability. (a and b) Knockdown of circEIF4G2 significantly suppressed HOS (a) and MG63 (b) cell proliferation using the CCK-8 assay. (c and d) Knockdown of circEIF4G2 significantly suppressed HOS (c) and MG63 (d) cell migration using the Transwell assay. (e and f) Knockdown of circEIF4G2 significantly suppressed HOS (e) and MG63 (f) cell migration using the Transwell assay.

**Figure 3:** Construction of circEIF4G2-mediated ceRNA networks in OS. A total of 5 miRNAs (hsa-miR-218-5p, hsa-miR-188-5p, hsa-miR-4465, hsa-miR-517-5p, and hsa-miR-525-5p) and 2187 mRNAs were included in the circEIF4G2-mediated ceRNA network in OS.

**Figure 4:** Bioinformatics analysis of circEIF4G2 in OS. (a) The GO analysis of circEIF4G2 in OS. (b) The KEGG pathway analysis of circEIF4G2 in OS.

**Figure 5:** CircEIF4G2 sponges miR-218. (a and b) Dual-luciferase reporter assays showed that miR-218 decreases the relative luciferase activity of the wild-type circEIF4G2 luciferase plasmid compared with the mutant in both HOS (a) and MG63 (b) cells. (c and d) Overexpression of miR-218 significantly suppressed HOS (c) and MG63 (d) cell proliferation using the CCK-8 assay. (e and f) Overexpression of miR-218 significantly suppressed HOS cell migration (e) and invasion (f) using the Transwell assay. (g and h) Overexpression of miR-218 significantly suppressed MG63 cell migration (g) and invasion (h) using the Transwell assay.

**Figure 6:** Silencing of miR-218 reverses the effects of circEIF4G2 knockdown in OS. (a and b) Silencing of miR-218 reversed the effects of decreased cell proliferation in circEIF4G2 knockdown HOS (a) and MG63 (b) cells. (c) Silencing of miR-218 reversed the effects of decreased cell migration in circEIF4G2 knockdown HOS cells. (d) Silencing of miR-218 reversed the effects of decreased cell invasion in circEIF4G2 knockdown HOS cells.

## Data Availability

All the date refer to bioinformatics analyses were stored at RegRNA 2.0 database (http://regrna2.mbc.nctu.edu.tw/index.html) and DAVID (https://david.ncifcrf.gov/).

## References

[1] Simpson E., Brown H. L. (2018). Understanding osteosarcomas. *Journal of the American Academy of Physician Assistants*.

[2] Liu X., Cui M. (2019). miRNA-98-5p inhibits the progression of osteosarcoma by regulating cell cycle via targeting CDC25A expression. *European Review for Medical and Pharmacological Sciences*.

[3] Jiang N., Wang X., Xie X. (2017). lncRNA DANCR promotes tumor progression and cancer stemness features in osteosarcoma by upregulating AXL via miR-33a-5p inhibition. *Cancer Letters*.

[4] Chen X., Zhang X., Cai H. (2020). Targeting USP9x/SOX2 axis contributes to the anti-osteosarcoma effect of neogambogic acid. *Cancer Letters*.

[5] He M., Shen P., Qiu C., Wang J. (2019). miR-627-3p inhibits osteosarcoma cell proliferation and metastasis by targeting PTN. *Aging*.

[6] Chen J., Yan C., Yu H., Zhen S., Yuan Q. (2019). miR-548d-3p inhibits osteosarcoma by downregulating <i>KRAS</i>. *Aging*.

[7] Yu X., Hu L., Li S. (2019). Long non-coding RNA Taurine upregulated gene 1 promotes osteosarcoma cell metastasis by mediating HIF-1*α* via miR-143-5p. *Cell Death & Disease*.

[8] Zhou Q., Hu T., Xu Y. (2020). Anticancer potential of TUG1 knockdown in cisplatin-resistant osteosarcoma through inhibition of MET/Akt signalling. *Journal of Drug Targeting*.

[9] Zhou R., Wu Y., Wang W. (2018). Circular RNAs (circRNAs) in cancer. *Cancer Letters*.

[10] Patop I. L., Kadener S. (2018). circRNAs in cancer. *Current Opinion in Genetics & Development*.

[11] Shang Q., Yang Z., Jia R., Ge S. (2019). The novel roles of circRNAs in human cancer. *Molecular Cancer*.

[12] Arnaiz E., Sole C., Manterola L., Iparraguirre L., Otaegui D., Lawrie C. H. (2019). circRNAs and cancer: biomarkers and master regulators. *Seminars in Cancer Biology*.

[13] Pan G., Hu T., Chen X., Zhang C. (2019). Upregulation of circMMP9 promotes osteosarcoma progression via targeting miR-1265/CHI3L1 axis. *Cancer Management and Research*.

[14] Zheng S., Qian Z., Jiang F. (2019). circRNA LRP6 promotes the development of osteosarcoma via negatively regulating KLF2 and APC levels. *American Journal of Translational Research*.

[15] Zhong Q., Huang J., Wei J., Wu R. (2019). Circular RNA CDR1as sponges miR-7-5p to enhance E2F3 stability and promote the growth of nasopharyngeal carcinoma. *Cancer Cell International*.

[16] Su Y., Lv X., Yin W. (2019). circRNA Cdr1as functions as a competitive endogenous RNA to promote hepatocellular carcinoma progression. *Aging (Albany NY)*.

[17] Zhao Z., Ji M., Wang Q., He N., Li Y. (2019). Circular RNA Cdr1as upregulates SCAI to suppress cisplatin resistance in ovarian cancer via miR-1270 suppression. *Mol Ther Nucleic Acids*.

[18] Zhang X., Yang D., Wei Y. (2018). Overexpressed CDR1as functions as an oncogene to promote the tumor progression via miR-7 in non-small-cell lung cancer. *Onco Targets Ther*.

[19] Xu B., Yang T., Wang Z., Zhang Y., Liu S., Shen M. (2018). circRNA CDR1as/miR-7 signals promote tumor growth of osteosarcoma with a potential therapeutic and diagnostic value. *Cancer Management and Research*.

[20] Xie X., Li Y. S., Xiao W. F. (2017). MicroRNA-379 inhibits the proliferation, migration and invasion of human osteosarcoma cells by targetting EIF4G2. *Bioscience Reports*.

[21] Kong Z., Wan X., Lu Y. (2020). Circular RNA circFOXO3 promotes prostate cancer progression through sponging miR-29a-3p. *Journal of Cellular and Molecular Medicine*.

[22] Chang T.-H., Huang H.-Y., Hsu J. B.-K., Weng S.-L., Horng J.-T., Huang H.-D. (2013). An enhanced computational platform for investigating the roles of regulatory RNA and for identifying functional RNA motifs. *BMC Bioinformatics*.

[23] Gradi A., Imataka H., Svitkin Y. V. (1998). A novel functional human eukaryotic translation initiation factor 4G. *Molecular and Cellular Biology*.

[24] Imataka H., Gradi A., Sonenberg N. (1998). A newly identified N-terminal amino acid sequence of human eIF4G binds poly(A)-binding protein and functions in poly(A)-dependent translation. *The EMBO Journal*.

[25] Ruggero D., Montanaro L., Ma L. (2004). The translation factor eIF-4E promotes tumor formation and cooperates with c-Myc in lymphomagenesis. *Nature Medicine*.

[26] Hao G. J., Hao H. J., Ding Y. H. (2017). Suppression of EIF4G2 by miR-379 potentiates the cisplatin chemosensitivity in nonsmall cell lung cancer cells. *FEBS Letters*.

[27] Gu C., Pan X., Wang R. (2016). Analysis of mutational and clinicopathologic characteristics of lung adenocarcinoma with clear cell component. *Oncotarget*.

[28] Gu C., Huang Z., Dai C. Prognostic analysis of limited resection versus lobectomy in stage IA small cell lung cancer patients based on the surveillance, epidemiology, and end results registry database. *Frontiers in Genetics*.

[29] Mao Y., Zhang L., Li Y. (2019). CircEIF4G2 modulates the malignant features of cervical cancer via the miR‑218/HOXA1 pathway. *Molecular Medicine Reports*.

[30] Li X. N., Wang Z. J., Ye C. X., Zhao B. C., Li Z. L., Yang Y. (2018). RNA sequencing reveals the expression profiles of circRNA and indicates that circDDX17 acts as a tumor suppressor in colorectal cancer. *Journal of Experimental & Clinical Cancer Research*.

[31] Wang W., Zhao H. F., Yao T. F., Gong H. (2019). Advanced development of ErbB family-targeted therapies in osteosarcoma treatment. *Investigational New Drugs*.

[32] Gill J., Geller D., Gorlick R. (2014). HER-2 involvement in osteosarcoma. *Advances in Experimental Medicine and Biology*.

[33] Sheng J., Yin M., Sun Z. (2017). SPC24 promotes osteosarcoma progression by increasing EGFR/MAPK signaling. *Oncotarget*.

[34] Rupaimoole R., Slack F. J. (2017). MicroRNA therapeutics: towards a new era for the management of cancer and other diseases. *Nature Reviews Drug Discovery*.

[35] Xue D., Wang H., Chen Y. (2019). Circ-AKT3 inhibits clear cell renal cell carcinoma metastasis via altering miR-296-3p/E-cadherin signals. *Molecular Cancer*.

[36] Zhang Y., Liu H., Li W. (2017). circRNA_100269 is downregulated in gastric cancer and suppresses tumor cell growth by targeting miR-630. *Aging (Albany NY)*.

[37] Zhang J., Liu H., Hou L. (2017). Circular RNA_LARP4 inhibits cell proliferation and invasion of gastric cancer by sponging miR-424-5p and regulating LATS1 expression. *Molecular Cancer*.

[38] Xuan C., Jin M., Gao Y. (2019). miR-218 suppresses the proliferation of osteosarcoma through downregulation of E2F2. *Oncology Letters*.

[39] Wang D. Z., Jing S. F., Hao S. B., Huang X. Y., Miao Q. T., Gao J. F. (2018). MiR-218 promotes apoptosis of U2OS osteosarcoma cells through targeting BIRC5. *European Review for Medical and Pharmacological Sciences*.

[40] Jin J., Cai L., Liu Z. M., Zhou X. S. (2013). miRNA-218 inhibits osteosarcoma cell migration and invasion by down-regulating of TIAM1, MMP2 and MMP9. *Asian Pacific Journal of Cancer Prevention*.

